The article "MicroRNA-124 Regulates the Proliferation of Colorectal Cancer Cells by Targeting iASPP" was retracted in 2023. Reasons: plagiarized text; overlap with other authors' work.

# MicroRNA-124 Regulates the Proliferation of Colorectal Cancer Cells by Targeting *iASPP*

**DOI:** 10.1155/2013/867537

**Published:** 2013-04-10

**Authors:** Kuijie Liu, Hua Zhao, Hongliang Yao, Sanlin Lei, Zhendong Lei, Tiegang Li, Haizhi Qi

**Affiliations:** Department of General Surgery, The Second Xiangya Hospital, Central South University, Changsha, Hunan 410011, China

## Abstract

MicroRNAs are a class of small, noncoding RNAs that function as critical regulators of gene expression by targeting mRNAs for translational repression or degradation. In this study, we demonstrate that expression of microRNA-124 (miR-124) is significantly downregulated in colorectal cancer tissues and cell lines, compared to the matched adjacent tissues. We identified and confirmed inhibitor of apoptosis-stimulating protein of p53 (*iASPP*) as a novel, direct target of miR-124 using target prediction algorithms and luciferase reporter gene assays. Overexpression of miR-124 suppressed iASPP protein expression, upregulated expression of the downstream signaling molecule nuclear factor-kappa B (NF-***κ***B), and attenuated cell viability, proliferation, and colony formation in SW480 and HT-29 colorectal cancer cells in vitro. Forced overexpression of *iASPP* partly rescued the inhibitory effect of miR-124 on SW480 and HT29 cell proliferation. Taken together, these findings shed light on the role and mechanism of action of miR-124, indicate that the miR-124/iASPP axis can regulate the proliferation of colorectal cancer cells, and suggest that miR-124 may serve as a potential therapeutic target for colorectal cancer.

## 1. Introduction

Colorectal cancer (CRC) still is the common cancer, the third leading cause of cancer deaths in the whole world [1], and generally has a very poor prognosis due to its high propensity for tumor invasion and migration. Although invasion and migration have been acknowledged as the most lethal attributes of solid tumors, knowledge of the molecular mechanisms underlying these processes is still limited.

Recently, growing evidence has supported cancer-related roles for microRNAs (miRNAs), a newly discovered class of small, noncoding RNAs which negatively regulate the expression of a variety of genes. MicroRNAs affect multiple cellular pathways through inducing the mechanism of RNA interference at the posttranscription level. Primary miRNAs (pri-miRNAs) are transcribed by RNA polymerase, then processed into smaller precursor hairpin structures (pre-miRNAs) in the nucleus, and exported to the cytoplasm. They are further processed by the nuclease Dicer to mature functional miRNAs approximately 21 nucleotides in length. Mature miRNAs induce mRNA degradation or inhibit translation by integrating into an RNA-inducing silencing complex (RISC) and binding to specific complementary sites within the 3′ untranslated regions (3′ UTR) of their target mRNAs [2–6]. Bioinformatic algorithms indicate that human miRNAs perhaps regulate up to 30% of all human genes, which represent the majority of cellular pathways [7, 8]. Due to the complicated combination relationships between miRNAs and mRNA 3′ UTRs, several online tools have been developed for miRNA target prediction. These resources are used to microRNA target predictions based on sequence complementarity, including TargetScan [5], PicTar [7], and TargetRank [8], which provide precise base pairing of the miRNA to the seed region and sequence conservation.

The article "MicroRNA-124 Regulates the Proliferation of Colorectal Cancer Cells by Targeting iASPP" was retracted in 2023. Reasons: plagiarized text; overlap with other authors' work.

Inhibitor of apoptosis stimulating protein of p53 (iASPP), also known as RelA-associated inhibitor (RAI), is one of the most ancient members of the ASPP protein family, and an evolutionarily conserved inhibitor of p53. As a binding partner, iASPP negatively regulates the RelA subunit (p65RelA) of the nuclear factor-kappa B (NF-*κ*B), which plays a pivotal role in the inflammatory response and apoptosis [9, 10]. Therefore, it is likely that the expression level or activity of iASPP would influence the availability of NF-*κ*B, and thus modify the regulation of cell growth. iASPP may serve as an independent prognostic marker of tumor proliferation in some other cancer types. Li et al. [11] reported that knockdown of iASPP significantly inhibited cell growth and proliferation in U251 cells. Zhang et al. [12] reported that the expression of iASPP in tumor tissues was higher than the adjacent tissues of prostate cancer. Downregulation of the expression of iASPP by shRNA inhibited proliferation and induced apoptosis of p53-defective prostate cancer cells. Existing data regarding the involvement of iASPP in tumor metastasis also suggests thatit may have potential as a therapeutic target [6, 13].

In order to identify novel microRNAs which could specifically target iASPP, several candidate microRNAs (miR-124, miR-506, miR-182, miR-19a, and miR-19b) were initially predicted by software analysis programme. We therefore challenged their expression in patient samples and also explored iASPP inhibition in colorectal cancer cells by introduction of exogenous miRNA expression. miR-124 expression was decreased significantly in CRC tissues compared to the adjacent normal colonic tissues in a panel of matched  tissues  from  17  CRC  patients. In the present study, we confirmed the regulatory relationship between miR-124, a known tumor-suppressive miRNA, and an oncogene, *iASPP*. We provide evidence that miR-124 can inhibit CRC cell proliferation, at least in part by targeting *iASPP*. Ectopic overexpression of miR-124 downregulated iASPP protein expression and upregulated NF-*κ*B protein expression. Force expression of iASPP rescued the effects of miR-124. These results provide novel insights into our understanding of the role and mechanism of miR-124 in the pathoetiology of CRC, which may provide a potential therapeutic strategy for treatment of CRC in the future.

The article "MicroRNA-124 Regulates the Proliferation of Colorectal Cancer Cells by Targeting iASPP" was retracted in 2023. Reasons: plagiarized text; overlap with other authors' work.

## 2. Materials and Methods

### 2.1. Tissue Samples, Cell Lines, and Cell Transfection

A total of 17 paired primary CRC tissues and the matched adjacent normal colonic epithelial tissues were collected. All samples were obtained from patients who underwent surgical resection at The Second Xiangya Hospital of Central South University (Changsha, China). The tissues were snap-frozen in liquid nitrogen, and then stored at −80°C. This project was approved by the Ethics Committee of The Second Xiangya Hospital of Central South University.

Human CRC cell lines, including SW480, SW620, and HT29 cells, were purchased from the American Type Culture Collection (Manassas, VA, USA) and cultured in RPMI-1640 medium (Invitrogen, Carlsbad, CA, USA) supplemented with 10% fetal bovine serum (Gibco, CA, USA) at 37°C in a humidified atmosphere with 5% CO_2_. Ectopic overexpression of miR-124 was achieved by transfection of miR-124 lentivirus (Genepharma, Shanghai, China) using Lipofectamine 2000 (Invitrogen). Overexpression of iASPP was achieved using an *iASPP* ORF-expressing clone (GeneCopoecia, Guangzhou, China). Cells were plated in 6-well plates or 96-well plates, transfected, incubated for 24 h or 48 h, and used for further assays or RNA/protein extraction.

### 2.2. Construction of miR-124 and iASPP shRNA Expressing Lentivirus Vectors

To generate lentivirus expressing mature miR-124, the pre-miRNA sequence was synthesized; a control scrambled construct (control RNAi) with no homology to the human genome was also created (AAT GTA CTG CGC GTG GAG A). The sequences were cloned into the *Hpa*I and *Xho*I sites of pGCSIL-GFP (GeneChem, Shanghai, China) to generate pGCSIL-GFP-miR-124 or pGCSIL-GFP-Ctr, respectively. Viral shRNA targeting *iASPP* was purchased from Auragene Bioscience Inc. (Changsha, China). 

### 2.3. Lentivirus Production, Titration, and Infection

To generate miR-124 or control lentivirus, the plasmids encoding miR-124 or the control scrambled sequence were cotransfected into 293T cells together with the plasmids pHelper1.0 and pHelper 2.0 (Genechem, Shanghai, China) which contain the elements required for virus packaging, using Lipofectamine 2000 (Invitrogen, CA, USA) according to the manufacturer's instructions. The culture supernatants containing lentivirus were harvested and concentrated by ultracentrifuge, and the viral titers were determined. To perform lentiviral infection, the target cells were plated at 40%–50% confluence and incubated overnight (16 h). On the day of infection, the culture medium was replaced with viral supernatant at an appropriate titer (1.5 mL/well), incubated at 37°C for 10 h, then the viral supernatant was replaced with fresh media. Forty-eight hours later, the infected cells were selected using puromycin (2 mg/mL). After 5 days of selection, shRNA knockdown efficiency was determined by real-time PCR and Western blot analysis.

The article "MicroRNA-124 Regulates the Proliferation of Colorectal Cancer Cells by Targeting iASPP" was retracted in 2023. Reasons: plagiarized text; overlap with other authors' work.

### 2.4. RNA Extraction and Quantitative Real-Time RT-PCR

Total RNA was extracted from 10–20 mg of tumor samples and from 30–40 mg of normal tissues. Samples were mechanically disrupted and simultaneously homogenized in the presence of QIAzol Lysis reagent (Qiagen, Valencia, CA, USA), using a Mikrodismembrator (Braun Biotech International, Melsungen, Germany). RNA was extracted using the miRNeasy Mini kit (Qiagen) according to the manufacturer's instructions.

Approximately 1.0 × 10^6^ SW480 or HT29 cells (uninfected or infected) were seeded into 6-well culture plates, cultured for 72 h, and harvested. Small RNAs (~200 nt) were isolated using the mirVanaTM PARIS TM Kit (Ambion, CA, USA) according to the manufacturer's instructions. 

For RT reactions, 1 mg of small RNAs was reverse transcribed with the miScript Reverse Transcription Kit (Qiagen, CA, USA) at 37°C for 60 min followed by a final incubation at 95°C for 5 min. miRNA real-time RT-PCR was carried out using the miScript SYBR Green PCR kit (Qiagen) on an CFX96 real-time PCR machine (Bio-Rad, Hercules, CA, USA). PCR was conducted at 95°C for 15 min, followed by 40 cycles of 94°C for 15 s, 55°C for 30 s, and 70°C for 30 s. The expression of each miRNA was normalized to U6 snRNA. 

Expression of *iASPP* mRNA was detected by quantitative real-time RT-PCR (qRT-PCR) using the standard SYBR Green RT-PCR Kit (Bio-Rad, CA, USA) according to the manufacturer's instructions. Briefly, total RNA was extracted from the cells using TRIzol reagent (Invitrogen) and cDNA was synthesized using the RevertAid First-Strand cDNA Synthesis kit (Fermentas, CA, USA, according to the manufacturer's protocol. Each cDNA sample was used as a template for PCR in triplicate with iQTM SYBR Green Supermix (Bio-Rad, CA, USA) by denaturation at 94°C for 1 min; 30 cycles of 94°C for 40 and 60°C for 40 s; followed by extension at 72°C for 6 min. The specific primer pairs were *iASPP* (107 bp), sense: 5′-GGC GGT GAA GGA GAT GAA C −3′; antisense: 5′-TGA TGA GGA AAT CCA CGA TAG AG-3′; **β*-actin* (202 bp) sense: 5′-GGC GGC ACC ACC ATG TAC CCT-3′; reverse: 5′-AGG GGC CGG ACT CGT CAT ACT-3′. The relative levels of *iASPP* mRNA were normalized to the internal control **β*-actin*. Relative gene expression was quantified using CFX Manager software (Bio-Rad, CA, USA) and expressed as percentage of control cells.

The article "MicroRNA-124 Regulates the Proliferation of Colorectal Cancer Cells by Targeting iASPP" was retracted in 2023. Reasons: plagiarized text; overlap with other authors' work.

### 2.5. Western Blotting

Cells cultured in 35 mm dishes were lysed in 0.2 mL lysis buffer (0.1% SDS, 1% NP-40, 50 mM HEPES, pH 7.4, 2 mM EDTA, 100 mM NaCl, 5 mM sodium orthovanadate, 40 *μ*M p-nitrophenyl phosphate and 1% protease inhibitor mixture set I (Calbiochem, USA). Lysates were centrifuged at 12,000 rpm for 15 min, the supernatants were collected, denatured, separated using 10% SDS-PAGE gels, and blotted onto polyvinylidene difluoride membranes. The membranes were blocked in 5% albumin from bovine serum (BSA) for 1.5 h at room temperature, then probed with 1 : 1000 diluted rabbit polyclonal iASPP and NF-*κ*B (p65) antibody (Abcam, MA, USA) at 4°C overnight, and the blots were subsequently incubated with HRP-conjugated secondary antibody (1 : 5000). Signals were visualized using ECL Substrates (Millipore, MA, USA). *β*-actin was used as an endogenous protein for normalization.

### 2.6. MTT Assay

Cell viability was evaluated using a modified MTT assay. The viability of SW480 or HT29 cells transfected with miR-124 or control was assessed at five time points (on days 1, 2, 3, 4, and 5) after seeding 2 × 10^3^ transfected cells/well into 96-well culture plates. Briefly, quantification of mitochondrial dehydrogenase activity was achieved via the enzymatic conversion of MTT (3-(4,5-dimethylthiazol-2-yl)-2,5-diphenyltetrazolium bromide; Sigma-Aldrich, MO, USA) to a colored formazan product. MTT (10 *μ*L, 10 mg/mL) was added to the cells, incubated for 4 h, and the reaction was terminated by removal of the supernatant and addition of 100 *μ*L DMSO to dissolve the formazan product. After 0.5 h, the optical density (OD) of each well was measured at 570 nm using a plate reader (ELx808 Bio-Tek Instruments, City, ST, USA).

### 2.7. BrdU Incorporation Assay

DNA synthesis in proliferating cells was determined by measuring 5-Bromo-2-deoxyUridine (BrdU) incorporation. BrdU assays were performed at 24 h and 48 h after transfecting SW480 or HT29 cells with miR-124 or control vector. The infected cells were seeded in 96-well culture plates at a density of 2 × 10^3^ cells/well, cultured for 24 h or 48 h, and incubated with a final concentration of 10 *μ*M BrdU (BD Pharmingen, San Diego, CA, USA) for 2 h to 24 h. At the end of the incubation period, the medium was removed, the cells were fixed for 30 min at RT, incubated with peroxidase-coupled anti-BrdU-antibody (Sigma-Aldrich) for 60 min at RT, washed three times with PBS, incubated with peroxidase substrate (tetramethylbenzidine) for 30 min, and the absorbance values were measured at 490 nm. Background BrdU immunofluorescence was determined in cells not exposed to BrdU but stained with the BrdU antibody.

The article "MicroRNA-124 Regulates the Proliferation of Colorectal Cancer Cells by Targeting iASPP" was retracted in 2023. Reasons: plagiarized text; overlap with other authors' work.

### 2.8. Colony Formation Assay

The effect of *iASPP* silencing on the colony formation ability of SW480 or HT29 cells was analyzed using the colony formation assay. SW480 or HT29 control, RNAi control, or *iASPP* RNAi cells were plated at 200 cells per well in 6-well culture plates and cultured in DMEM containing 10% FBS at 37°C and 5% CO_2_ for 2 weeks. The cell colonies were washed twice with PBS, fixed with 4% paraformaldehyde (PFA) for 15 min, stained with Gimsa for 20 min, and washed twice with ddH2O. Individual clones with more than 50 cells were counted. 

### 2.9.  3′ UTR Luciferase Reporter Assay

UTR luciferase reporter assays were performed in human embryonic kidney 293 (HEK293) cells. Vectors based on pMIR-REPORT harboring the wild-type (WT) 350 bp fragment of the *iASPP* 3′ UTR, or the same fragment in which the miR-124 binding site (199–194) was mutated (MUT), were inserted downstream of the luciferase reporter gene stop codon in pMIR-REPORT using *Hind*III and *Spe*I. The cells were cotransfected with (1) miR-124 lentivirus or miR-67-negative-control lentivirus (50 nM), (2) pMIR-REPORT vectors containing the WT or MUT miR-124 binding sites (400 ng), and (3) pRL-SV40 (Promega, Sunnyvale, CA, USA) expressing Renilla luciferase (400 ng) for normalization of transfection efficiency. Cells were grown in high-glucose DMEM supplemented with 10% fetal bovine serum, and luciferase activities were measured at 48 h after transfection using the Dual-Luciferase Reporter Assay System (Promega).

### 2.10. Statistical Analysis

Data were expressed as mean ± SD of three independent experiments and processed using SPSS 17.0 statistical software (SPSS, Chicago, IL, USA). The expression of miR-124 in CRC tissues and the paired adjacent normal colonic tissues were compared using Wilcoxon's paired test. The differences between groups in the migration and invasion assays were evaluated using the one-way ANOVA. *P* values of < 0.05 were considered statistically significant.

## 3. Results

### 3.1. miR-124 Is Frequently Downregulated in CRC Tissues and Cell Lines

Targetscan and microRNA.org [14, 15] predicted that miR-124, miR-506, miR-182, miR-19a, and miR-19b could bind to and target the *iASPP* 3′ UTR. In the present study, we first examined the expression levels of these miRNAs in clinical samples of CRC tissues and matched normal tissues using qPCR. Expression of miR-214 was found to be downregulated in tumor tissues compared with the matched normal tissues in 14/17 (82.3%) of samples. In 70.6%, (12/17) of samples, miR-506 was found to be downregulated. Figures 1(a) and 1(b) show the mean expression levels of miR-214 and miR-506, which were significantly lower in tumor tissues than in matched normal tissues. On the other hand, the expression levels of miR-182, miR-19a, and miR-19b were not significantly different between tumor and matched normal tissues (Figures 1(c)–1(e)). In addition, miR-124 was also expressed at significantly lower levels in the three human CRC cell lines compared to the normal human colon cell line (Figure 1(f)).

The article "MicroRNA-124 Regulates the Proliferation of Colorectal Cancer Cells by Targeting iASPP" was retracted in 2023. Reasons: plagiarized text; overlap with other authors' work.

### 3.2. iASPP mRNA Is a Direct Target of miR-124

To determine whether the 3′-UTR of iASPP mRNA is a functional target of miR-214 in CRC cells, we created a WT-*iASPP* 3′ UTR luciferase reporter vector (WT-iASPP), as well as a MUT-*iASPP* 3′ UTR luciferase reporter vector (MUT-iASPP) by sequentially mutating the predicted 8-base pair miR-124 binding site in the *iASPP* 3′ UTR (Figure 2(a)). We co-transfected the WT-iASPP vector and miR-124 lentivirus or a scrambled control into HEK293 cells. The luciferase activity of the *iASPP* 3′ UTR luciferase reporter vector was significantly reduced in miR-124 transfected cells, compared to scrambled control cells (Figure 2(b)). Moreover, miR-124-mediated repression of *iASPP* 3′ UTR luciferase reporter activity was abolished by mutation of the putative miR-24 binding site in the *iASPP* 3′ UTR (Figure 2(b)).

### 3.3. Knockdown of iASPP or Overexpression of miR-124 Inhibit iASPP Expression and Increases NF-*κ*B (p65) Expression

We infected SW480 or HT29 cells with miR-124 and miR-scramble lentivirus, *iASPP* shRNA or shRNA-control lentivirus. Quantitative PCR showed that, at 96 h after transfection, miR-124 was significantly overexpressed in SW480 or HT29 cells infected with miR-124 lentivirus, compared to cells infected with the scrambled control lentivirus (Figure 3(a)). Overexpression of miR-124 or knockdown of *iASPP* using shRNA both led to a moderate decrease in *iASPP* mRNA expression in SW480 or HT29 cells (Figure 3(b)), suggesting that *iASPP *is potentially regulated by miR-124. These results indicated that miR-124 can transcriptionally regulate and inhibit iASPP expression. Additionally, Western blotting demonstrated that infection of miR-124 lentivirus or *iASPP* shRNA reduced iASPP protein expression (Figure 3(c)) and increased NF-*κ*B (p65) protein expression (Figure 3(d)). These results suggest that overexpression of miR-124 upregulated the expression of NF-*κ*B (p65), at least in part, by reducing the expression of iASPP.

The article "MicroRNA-124 Regulates the Proliferation of Colorectal Cancer Cells by Targeting iASPP" was retracted in 2023. Reasons: plagiarized text; overlap with other authors' work.

### 3.4. Overexpression of miR-124 or iASPP shRNA Attenuate CRC Cell Proliferation and Colony Formation

It has been reported that NF-*κ*B played a role in the cell proliferation and apoptosis [12]. To investigate if miR-124 can regulate CRC cell viability by targeting *iASPP *and upregulating NF-*κ*B, we transfected miR-124 lentivirus, control lentivirus, *iASPP* shRNA or shRNA-control into SW480 or HT29 cells, and performed the MTT assay. Overexpression of miR-124 or knockdown of *iASPP* significantly inhibited SW480 or HT29 cell viability, compared to cells transfected with scrambled control lentivirus (Figure 4(a)). Transfection of miR-124 lentivirus or *iASPP* shRNA also significantly suppressed SW480 or HT29 cell proliferation compared to the scramble control lentivirus, as indicated by the BrdU incorporation assay (Figure 4(b)). The colony formation assay indicated that cells transfected with *iASPP* shRNA (10%) or miR-124 lentivirus (30%) formed significantly lower numbers of colonies than shRNA-control-infected cells (100%; Figures 4(c) and 4(d)). These results suggest that overexpression of miR-124 attenuated cell proliferation by downregulating *iASPP* signaling.

### 3.5. Forced Expression of iASPP Restores the Effects of miR-124 in CRC Cells

As shown above, *iASPP* is a direct target gene of miR-124. Therefore, we wondered whether forced overexpression of iASPP could reverse miR-124-induced upregulation of NF-*κ*B (p65). An iASPP ORF-expressing plasmid was transfected into miR-124- or miR-SCR-expressing cells. As shown in Figure 5, the reduced expression of iASPP in miR-124-overexpressing cells was rescued by the introduction of *iASPP* cDNA. Similarly, ectopic overexpression of iASPP also prevented miR-124-induced NF-*κ*B (p65) upregulation in SW480 or HT29 cells, confirming that miR-124 upregulates NF-*κ*B (p65) by targeting *iASPP *mRNA.

## 4. Discussion

In this research, we identified and confirmed that *iASPP* is a target gene of human miR-124. A luciferase reporter assay validated the binding and repressive effects of miR-124 on the *iASPP* 3′-UTR in HEK293 cells. Additionally, qPCR demonstrated that miR-124 is downregulated in CRC cell lines and tumor tissues. A shRNA targeting *iASPP*, or overexpression of miR-124, downregulated the expression of iASPP and reduced the viability, proliferation, and colony formation ability of the CRC cancer cell line SW480 or HT29. In addition, overexpression of miR-124 downregulated the expression of iASPP and upregulated the expression of NF-*κ*B (p65), and overexpression of iASPP inhibited the ability of miR-124 to upregulate NF-*κ*B (p65) expression. 

The article "MicroRNA-124 Regulates the Proliferation of Colorectal Cancer Cells by Targeting iASPP" was retracted in 2023. Reasons: plagiarized text; overlap with other authors' work.

These results are consistent with research on leukemia, breast cancer, and nonsmall cell lung cancer, which identified that iASPP is expressed at high levels [16]. Additionally, genotype mapping of tissues from breast cancer patients suggested that iASPP might act to regulate the p53 and NF-*κ*B pathway, and therefore control the growth of cancer cells [17]. It was originally described as RelA-associated inhibitor (RAI), which binds to the NF-*κ*B subunit p65 (RelA) and inhibits its transcriptional activity [18–21]. This evidence suggests that altered regulation of iASPP may be involved in tumorigenesis. 

Recent studies found that the expression of iASPP in carcinoma tissues was higher than the normal colonic tissues from the same patients [22–24]. Knockdown of iASPP significantly inhibited cell proliferation and induced G0/G1 cell cycle arrest in U251 cells by regulating expression of p21Waf1/Cip1 and cyclin D1 [25]. Downregulation of iASPP in human hepatocellular carcinoma cells inhibits cell proliferation and tumor growth [26]. iASPP is important for bladder cancer cell proliferation [27]. These suggested that iASPP played an important role in cancer cell proliferation. However, it is unclear what cell signals iASPP directly regulated in cancer cell proliferation. It was reported that iASPP may maintain epithelial homeostasis by binding and inhibiting the activity of p65RelA [28]. Future genetic studies are needed to test whether iASPP as a key player in epithelial stratification, a function that is achieved through its ability to bind and inhibit p63's activities and suppress cellular senescence and terminal differentiation [9].

Here, we demonstrated that overexpression of miR-124 leads to upregulation of NF-*κ*B, due to downregulation of the miR-124 target gene *iASPP*. Forced overexpression of miR-124 also attenuated SW480 or HT29 cell viability, proliferation, and colony formation. These findings indicate a novel role and mechanism of action for miR-124 in tumors and suggest that miR-124 may provide a potential target for cancer therapy.

miR-124 has been reported to play a role in glioblastoma differentiation, especially when intracellular growth factors are absent [29]. Likewise, miR-124 is upregulated in SW480 or HT29 cells, which can undergo androgen-independent growth in vitro [30]. It is possible that an intrinsic mechanism connects growth factor depletion and miR-124-regulated cell growth; this hypothesis requires further investigation in vivo.

In summary, we identified that miR-124 inhibits CRC cell viability, proliferation, and colony formation through targeting *iASPP*; these effects were due, at least in part, to upregulation of NF-*κ*B. The miR-124/iASPP axis identified in this study may play a vital role in regulating the proliferation of CRC cells and may provide a potential diagnostic and therapeutic target for CRC.

The article "MicroRNA-124 Regulates the Proliferation of Colorectal Cancer Cells by Targeting iASPP" was retracted in 2023. Reasons: plagiarized text; overlap with other authors' work.

## Figures and Tables

**Figure 1:** miR-124 is downregulated in both primary CRC tissues and CRC cell lines. The expression of miRNAs in the CRC tissues and the matched normal tissues was detected by qRT-PCR and normalized to that of U6. Results showed that the expression of miR-124 (a) and miR-506 (b) were significant decreased in tumor tissue compared with the matched normal tissue; while there was no significantly difference in the expression of miR-182 (c), miR-19a (d), and miR-19b (e) between the two groups. Data are presented as individual samples (*n* = 17) with the line indicating the mean level. (f) miR-124 was expressed at significantly lower levels in three CRC cell lines in comparison with normal colonic mucosa pooled from three healthy individuals. The figure is representative of three experiments with similar results.

**Figure 2:** miR-124 directly targets *iASPP* by binding to its 3′ UTR. (a) The predicted miR-124 binding site within the 3′ UTR of *iASPP* and the mutated version generated by site mutagenesis are shown. (b) Repression of wild-type *iASPP* 3′ UTR luciferase reporter gene activity by miR-124 (**P < 0.01); miR-124 had no effect on the luciferase activity of the mutated *iASPP* 3′ UTR reporter vector compared to control HEK293 cells or cell transfected with scrambled miR lentivirus (without miR-124) (miR-SRC).

**Figure 3:** Knockdown of *iASPP* or overexpression of miR-124 inhibits iASPP expression and increases NF-*κ*B(p65) expression. SW480 or HT29 or HT29 cells were infected with scrambled miR lentivirus (without miR-124) (miR-SRC), miR-124 lentivirus, *iASPP* shRNA, or control shRNA, lentivirus. (a) Real-time PCR analysis of miR-124 and U6 expression. (b) Real-time PCR quantification of *iASPP* mRNA expression; **P < 0.01 compared to SW480 or HT29 or HT29 cells transfected with scrambled miR-124 lentivirus (miR-SRC) or control shRNA lentivirus. (c) Western blot of iASPP protein expression. Expression of iASPP was inhibited by both *iASPP* shRNA and miR-124, compared to SW480 or HT29 or HT29 cells expressing Con-shRNA or miR-SCR. (d) Western blot of NF-*κ*B(p65) protein expression. Expression of NF-*κ*B(p65) was increased by both *iASPP* shRNA and miR-124, compared to SW480 or HT29 or HT29 cells expressing Con-shRNA or miR-SCR. The figure is representative of three experiments with similar results.

**Figure 4:** Effects of miR-124 and iASPP on the viability, proliferation, and clone forming ability of SW480 or HT29 or HT29 cells. SW480 or HT29 cells were transfected with scrambled miR lentivirus (without miR-124) (miR-SRC), miR-124 lentivirus, *iASPP* shRNA, or control shRNA. (a) MTT cell proliferation assay. Ectopic overexpression of miR-124 using an miR-124 lentivirus or *iASPP* shRNA significantly reduced the proliferation of SW480 or HT29 cells, compared to NC (**P < 0.01) (b) Cell viability, as determined by the BrdU incorporation assay. (c) Colony formation assay. Cells were seeded in soft agar as described in Section 2. (d) Number of colonies at two weeks after seeding. The figure is representative of three experiments with similar results.

The article "MicroRNA-124 Regulates the Proliferation of Colorectal Cancer Cells by Targeting iASPP" was retracted in 2023. Reasons: plagiarized text; overlap with other authors' work.

**Figure 5:** Overexpression of iASPP inhibits the effects of miR-124 on iASPP and NF-*κ*B(p65) expression. SW480 or HT29 cells stably expressing miR-SCR or miR-124 were transfected with *iASPP* ORF-expressing plasmid. After 48 h, the levels of specific proteins were analyzed by immunoblotting, and the band intensities were quantified using Image-Pro Plus and normalized to *β*-actin. (a and c) Overexpression of iASPP increased iASPP protein expression. (b and d) Overexpression of iASPP decreased NF-*κ*B(p65) protein expression; **P < 0.01.
